# Progress of Statin Therapy in the Treatment of Idiopathic Pulmonary Fibrosis

This article has been retracted.

**DOI:** 10.1155/2022/6197219

**Published:** 2022-03-19

**Authors:** Leiya Kou, Pei Kou, Guangwei Luo, Shuang Wei

**Affiliations:** ^1^Department of Respiratory Medicine, Wuhan No. 1 Hospital, Wuhan 430022, China; ^2^Hubei University of Chinese Medicine, Wuhan 430065, China; ^3^Department of Medical Record, Wuhan No. 1 Hospital, Wuhan 430022, China; ^4^Department of Respiratory and Critical Care Medicine, Tongji Hospital Tongji Medical College Huazhong University of Science and Technology, Wuhan 430030, China

## Abstract

Idiopathic pulmonary fibrosis (IPF) is a type of interstitial lung disease (ILD) characterized by the proliferation of fibroblasts and aberrant accumulation of extracellular matrix. These changes are accompanied by structural destruction of the lung tissue and the progressive decline of pulmonary function. In the past few decades, researchers have investigated the pathogenesis of IPF and sought a therapeutic approach for its treatment. Some studies have shown that the occurrence of IPF is related to pulmonary inflammatory injury; however, its specific etiology and pathogenesis remain unknown, and no effective treatment, with the exception of lung transplantation, has been identified yet. Several basic science and clinical studies in recent years have shown that statins, the traditional lipid-lowering drugs, exert significant antifibrotic effects, which can delay the progression of IPF and impairment of pulmonary function. This article is aimed at summarizing the current understanding of the pathogenesis of IPF, the progress of research on the use of statins in IPF models and clinical trials, and its main molecular targets.

## 1. Introduction

Idiopathic pulmonary fibrosis (IPF) is a chronic, progressive, and fibrotic interstitial lung disease (ILD) characterized by alveolar epithelial cell damage and abnormal repair mechanisms [1]. IPF is a fatal lung disease that affects middle-aged and elderly individuals [2]. In recent years, the incidence and prevalence of IPF have increased as the methodology for its diagnosis has been optimized and the average age of the population has increased [3]. The etiology of IPF remains unclear; however, the risk factors include smoking history, exposure to metallic dust, viral infection, and traits that are genetically inherited. The main symptoms of IPF include dyspnea and cough, which can manifest 4–5 years before the diagnosis of IPF [4]. Most patients with IPF demonstrate a gradual and progressive worsening of pulmonary function over time. The prognosis of IPF is poor, with an average survival of 3–5 years after diagnosis if left untreated [5]. Some patients with IPF may experience an acute deterioration of respiratory function over a short period of time; this acute exacerbation of IPF (AE-IPF) is the cause of death in such patients [6].

Pirfenidone and nintedanib have been approved by the US Food and Drug Administration in the treatment of IPF; they are efficacious in delaying the decline of lung function and reducing mortality [7]. However, the high cost and side effects associated with these drugs limit their clinical applicability. IPF is irreversible and eventually develops into end-stage lung disease even with the administration of these drugs. Therefore, lung transplantation is the only effective and feasible treatment modality that can prolong the life span and improve the quality of life in patients with IPF [8]. The scarcity of organs, high cost of surgery, and risk of immune reactions prevent lung transplantation from being used as the first-line treatment option for most patients with IPF, most of whom are still treated with medication and oxygen therapy.

Statins, which act as 3-hydroxy-3-methylglutaryl-coenzyme A (HMG-CoA) reductase inhibitors, are widely used to lower lipid levels by inhibiting cholesterol synthesis. They are the first-line treatment option for hyperlipidemia and coronary heart disease. In recent years, a growing body of research has demonstrated that statins can suppress inflammatory responses, reduce the expression of cytokines, attenuate oxidative stress (OS), inhibit myofibroblast differentiation, prevent pulmonary parenchyma remodeling, and block the key processes associated with fibrosis. Furthermore, several clinical studies have reported that statins could play an active role in the treatment of IPF, which may delay the decline of lung function and reduce mortality in patients with the disease. In this review, we focus on the progress of research studies investigating the use of statins in models of IPF and clinical trials, as well as the main molecular targets of the drugs, to provide a theoretical basis for the clinical application of this class of pharmacological agents.

## 2. Pathogenesis of IPF

### 2.1. The Role of Inflammatory Cells and Cytokines in the Pathogenesis of IPF

The etiology of IPF is unclear, and its pathogenesis has not been fully elucidated; however, there is sufficient evidence to demonstrate that the disease is related to inflammatory injury of the immune system, mediated by a variety of signaling pathways [9]. Some genetic studies conducted in recent years suggest that genetic predisposition may play a role in the development of IPF. Some have also shown that derangement of pulmonary surfactants or related components and alveolar collapse are common findings in patients with IPF [10]. Type II alveolar epithelial cells (AECIIs) are special secretory cells capable of producing and secreting large quantities of surfactants; therefore, they are more vulnerable to endoplasmic reticulum (ER) stress [11]. Mutations in the surfactant proteins due to ER stress chronically damage various cell types and tissues, promoting apoptosis of AECIIs [11]. The lungs have physiological repair functions that are initiated following tissue injury, and the repair and proliferation of normal AECs depend on the proliferation and differentiation of AECIIs. However, factors such as genetic predisposition, infection, or air pollution can injure AECs, resulting in dysfunction of their repair mechanisms [12], which regulates fibroblasts and promotes their differentiation through connective tissue growth factor (CTGF) and transforming growth factor beta (TGF-*β*) [13]. Conversely, fibroblasts produce angiotensin II and reactive oxygen species (ROS) to damage epithelial cells, and their interactions promote pulmonary fibrosis [13].

In the histologic analysis of IPF patients, inflammation was the most common histological feature, observed in approximately 25% of patients with IPF [14]. Following lung injury, AECs release inflammatory mediators, growth factors, and chemokines, resulting in the accumulation of neutrophils, macrophages, and lymphocytes at the site of injury. The functional phenotypes of macrophages generated by microenvironmental changes are diverse. There are two major macrophage phenotypes, including classically activated macrophages (M1) and selectively activated macrophages (M2). Several studies have shown that in the inflammatory stage, M1 macrophages produce nitric oxide (NO) through the inducible nitric oxide synthase (iNOS) and can also release cytokines such as interleukin-12 (IL-12), tumor necrosis factor alpha (TNF-*α*), and interleukin-1*β* (IL-1*β*) to combat pathogens [15]. M2 macrophages can produce profibrotic mediators, such as TGF-*β*, which can induce epithelial-mesenchymal transformation (EMT) through TGF-*β*/Smad2 signaling pathway and promote the proliferation of fibroblasts [16]. The study found that in a mouse model of bleomycin-induced pulmonary fibrosis, M2 macrophages were more recruited in lung tissue and they promoted the differentiation of myofibroblasts of lung resident mesenchymal stem cells [17]. TNF-*α*, which is produced by macrophages, is a proinflammatory factor that is closely related to the pathogenesis of IPF [18]. Studies have shown that TNF-*α* can inhibit the role of fibrogenic macrophages, thereby slowing the progression of fibrosis and promoting the degradation of fibrotic lesions [19]. However, TNF-*α* has been shown to activate the nuclear factor kappa B (NF-*κ*B) transcription factor, leading to myofibroblast differentiation of lung resident mesenchymal stem cells, which ultimately contributes to the deterioration of pulmonary fibrosis in the murine model of bleomycin-induced pulmonary fibrosis [20]. Interleukin 8 (IL-8), a cytokine secreted by macrophages, can also be produced by fibroblasts under appropriate stimulation conditions, leading to the activation or recruitment of neutrophils in lung tissue [21]. Immunohistochemical analysis of tissues collected during lung biopsy revealed numerous neutrophils infiltrating the lung parenchyma in patients with IPF [22]. Neutrophil elastase (NE) is one of the most important proteases released by neutrophils which can promote fibroblast proliferation and myofibroblast differentiation, which is a driver of pulmonary fibrosis, and is also associated with its severity [23]. Animal studies have shown that NE deficiency inhibits bleomycin-induced pulmonary fibrosis in mice, which is associated with inadequate activation of TGF-*β* [24]. One study demonstrated the accumulation of lymphocytes in the lung tissues of patients with IPF, even in those with end-stage disease [25]. IL-13 can induce fibrosis and is mostly secreted by T helper 2 cells (Th2). IL-13 levels were shown to be significantly increased in the bronchial epithelium and macrophages of patients with IPF [26], and the cytokines can activate the activator protein 1 (AP-1) transcription factor by interacting with the IL-13*α*2 receptor, thereby inducing the production of TGF-*β* in the alveolar macrophages [27]. IL-13 can also directly promote the proliferation of fibroblasts and collagen deposition to induce a fibrogenic response [28]. Mast cells are widely distributed around microvessels in the skin and visceral mucosa, secreting various cytokines and participating in immune regulation. Mechanical stress-induced mast cell degranulation activates the TGF-*β*1 signaling pathway, and the number of mast cells has been found to increase in pulmonary fibrosis and be positively correlated with disease severity [29].

Inflammatory cells and cytokines play an important role in pulmonary fibrosis. It is believed that damage to and abnormal repair of AECs are the basis of IPF. During lung tissue repair, normal reepithelialization cannot occur, resulting in alveolar injury. During this process, inflammatory cells aggregate and cytokine secretion increase, mediating various factors leading to pulmonary fibrosis.

### 2.2. The Role of TGF-*β* in the Pathogenesis of IPF

TGF-*β* is a multifunctional cytokine that regulates cell growth and differentiation and induces fibrosis and scar formation [30]. TGF-*β* is produced by a variety of cell types in the lung tissue, including alveolar macrophages, AECs, fibroblasts, and myofibroblasts, and it is temporarily stored in the ECM [31–33]. TGF-*β* is an important factor in the regulation of cellular activities; however, the pathway through which TGF-*β* becomes activated is not well understood, although it has been reported to be associated with certain conditions, including an acidic environment [34] and the presence of ROS [35] and integrins (*α*v*β*5 and *α*v*β*6) [36]. TGF-*β* receptors, including TGF-*β* receptors of type I (T*β*R-I), type II (T*β*R-II), and type III (T*β*R-III), are expressed in almost all tissues, although only the former two subtypes are involved in cell signaling [37]. TGF-*β* is activated by the large latent complex (LLC), which comprises latent transforming growth factor *β* binding proteins (LTBPs) and latency-associated peptide (LAP) before binding to its respective receptors. TGF-*β* recruits T*β*R-I into the glycine-serine-rich (GS) domain, where activated T*β*R-I phosphorylates its downstream targets after binding to T*β*R-II. Smad proteins, which are important regulatory molecules of the TGF-*β* superfamily of signaling proteins, are the downstream transmembrane receptors of TGF-*β* that are precisely regulated at different levels [38]. Activated TGF-*β* binds to the receptors on the surface of the cell membranes of fibroblasts and phosphorylates Smad2/3 proteins that bind to Smad4. Subsequently, the Smad complex translocates into the nucleus, acting as a marker of activation of the Smad2/3 signaling pathway, thereby regulating and driving EMT and the deposition of ECM [39–41].

In addition, TGF-*β* signal transduction could also affect Smad-independent signaling pathways, including those involving extracellular signal-regulated kinase (ERK), c-Jun N-terminal kinase (JNK), and p38 mitogen-activated protein kinase (MAPK). TGF-*β* is activated by binding to T*β*R-I; it then recruits and phosphorylates the ShcA domain on tyrosine and serine residues to induce the formation of the ShcA/growth factor receptor-bound protein 2 (Grb2)/Son of Sevenless (Sos) complex and further activates the Ras-Raf-MEK-ERK1/2 signaling pathway [42]. TGF-*β*-activated kinase 1 (TAK1), a member of the MAP kinase 3 (MAP3K) gene family, is activated by binding to TAK1 binding protein 1 (TAB1) and has been confirmed to be involved in the TGF-*β* signaling pathway. The activation of TGF-*β* promotes TGF-*β*-induced expression of collagen and the differentiation of fibroblasts through either the TAK1/TAB1-MKK3-p38 MAPK or TAK1/TAB1-MKK4-JNK signaling pathway [43, 44].

CTGF is an effective profibrotic mediator capable of inducing the proliferation of fibroblasts and the secretion of ECM, driving tissue fibrosis alongside TGF-*β* [45]. During lung tissue injury and repair processes, fibroblasts are generated and accompanied by lung tissue remodeling, which inactivates the Hippo signaling pathway and results in the translocation of Yes-associated protein (YAP) and transcriptional coactivator with PDZ-binding motif (TAZ) into the nucleus, activating the expression of CTGF (the target gene of the Hippo signaling pathway) and TGF-*β*, mediating fibroblast activation and ECM synthesis. Researchers have found high expression levels of YAP/TAZ in the nuclei of fibroblasts in the lung tissues of patients with IPF [46, 47]. Under the normal physiological conditions in cells, the Hippo signaling pathway mediates YAP phosphorylation through mammalian Ste20-like kinases 1/2 (MST1/2) and large tumor suppressor 1/2 (LATS1/2), which can cause YAP to remain in the cytoplasm for degradation [46].

Upon stimulation by factors released from the inflammatory cells, mast cells degranulate and activate TGF-*β* and *α*-smooth muscle actin (*α*-SMA), inducing the proliferation and activation of fibroblasts. In addition, fibroblasts can produce stem cell factors and nourish mast cells, which are processes that play a role in tissue fibrosis [29]. Fibroblast-specific protein 1 (FSP1), a fibroblast marker, is produced and secreted by macrophages of the M2 phenotype, which promotes the proliferation and activation of fibroblasts [48]. In a mouse model of bleomycin-induced pulmonary fibrosis, reduced expression of peroxisome proliferator-activated receptor gamma (PPAR-*γ*) was observed in AECs and alveolar macrophages of the lung tissues [49]. The mechanism by which low PPAR-*γ* expression leads to pulmonary fibrosis remains unclear, and PPAR-*γ* activation can inhibit TGF-*β*-induced transformation of fibroblasts into myofibroblasts as well as the deposition of ECM [50].

As mentioned above, TGF-*β* is a pleiotropic cytokine that binds to receptors to regulate cell proliferation, differentiation, and apoptosis, and it plays an important role in ECM synthesis and trauma repair. In summary, TGF-*β* activates Smad and Smad-independent signaling pathways, leading to fibroblast proliferation and excessive accumulation of ECM, which causes pulmonary fibrosis (see Figure 1).

### 2.3. The Role of ROS in the Pathogenesis of IPF

ROS play an important role in the progression of pulmonary fibrosis in animal models and patients with IPF [51, 52]. As early as 1987, Cantin et al. found that the amount of superoxide and hydrogen peroxide spontaneously released from the cells of patients with IPF was significantly higher than the levels released from normal cells [53]. Beeh et al. observed low levels of glutathione (GSH) in the sputum and plasma of patients with IPF [54]. GSH is an antioxidant that can help eliminate ROS to maintain homeostasis in organisms. It has been found that the main sources of ROS are derived from environmental toxins (such as exposure to ultraviolet light and tobacco), radiation, pharmaceutical agents (such as in the bleomycin-induced pulmonary fibrosis model in animals), and factors released from activated inflammatory cells [55]. The mitochondria are important organelles for generating cellular energy and are the main site of oxidative stress regulation in cells, and they are an important source of ROS production [56]. In addition to the generation of ROS by mitochondria, nicotinamide adenine dinucleotide phosphate (NADPH) oxidase (NOX) is an enzyme that is specially used to produce ROS, and a close relationship has been demonstrated between IPF and NOX, mainly NOX4. In a bleomycin-induced mouse model of acute lung injury, NOX4 expression increased significantly from day 7 to day 28, which could be inhibited by the knockdown of NOX4 using small interfering RNA [57]. However, the lung tissues of the NOX4-deficient mice were mostly normal, with only a small accumulation of myofibroblasts [58]. As early as 2001, Wassmann et al. found that atorvastatin could inhibit NOX activity, reduce vascular ROS production, and improve vascular endothelial cell dysfunction in spontaneously hypertensive rats [59]. Thus, the inhibition of NOX expression and ROS production represents a significant advance in the antifibrotic treatment of IPF.

Other studies found that TGF-*β*-induced gene expression in primary normal human lung fibroblasts requires the participation of ROS [60], and ROS can stimulate the differentiation of fibroblasts into myofibroblasts, which is important in the pathogenesis of IPF [61]. As described above, various cells in the body secrete inactive TGF-*β* (also known as LAP); ROS can directly oxidize LAP to activate TGF-*β*, and TGF-*β* can also induce the production of ROS [62]. This interaction between TGF-*β* and ROS is one of the causes of pulmonary fibrosis. It has been reported that destruction of the integrity of the epithelial barrier and apoptosis of AECIIs are important events in the pathogenesis of IPF, and these processes may be related to the continuous release of ROS [58]. *In vivo*, ROS can directly bind to lipids on cell membranes, causing oxidation reactions that eventually lead to lipid peroxidation. The end product of lipid peroxidation is malondialdehyde (MDA), which damages mitochondrial DNA (mtDNA) and induces apoptosis [63]. MDA content is an important parameter that reflects the potential antioxidant capacity of the body and can indirectly reflect the degree of peroxidative damage to tissues and cells [64]. In addition, several studies have found that MDA content is significantly increased in models of bleomycin-induced pulmonary fibrosis in rats [65–67], suggesting that oxidative damage caused by the imbalance between redox reactions plays an important role in the pathogenesis of IPF. At excessive levels, ROS target the mitochondria, inducing mitochondrial permeability transition pore (MPTP) opening and the release of cytochrome c, which can directly or indirectly participate in the activation of caspases and the induction of cellular apoptosis [68]. One study found upregulation of proapoptotic factors p53, p21, B-cell lymphoma 2-associated X protein (Bax), and caspase-3 and downregulation of the expression of antiapoptotic factor B-cell lymphoma 2 (Bcl-2) in the bronchial cells and AECs of patients with IPF [69]. Another study reported increased apoptosis in human A549 cells and rat primary isolated AECIIs treated with asbestos, which was associated with enhanced ROS-related ER stress and Ca^2+^ release [70]. Some studies have shown that ROS can mediate the p38, JNK, and ERK signaling pathways and lead to apoptosis of lung epithelial cells [71, 72].

There is evidence to show that p38 MAPK is activated in response to the fibrosis induced by single-walled carbon nanotubes, a process that requires the participation of ROS [73]. The same study also found that this profibrotic substance induced TGF-*β* activation, upregulated collagen expression, and induced fibrosis in the lung fibroblasts through the ROS-mediated p38 MAPK signaling [73].

In addition to their lipid-lowering properties, statins have antioxidative properties. For example, many studies have confirmed that statins can inhibit NOX activity and reduce ROS production [74–76]. ERK, a member of the MAPK family, mediates a variety of cellular processes, including those related to cell growth, differentiation, and death. The ERK signaling pathway, especially ERK1/2, is closely related to the fibroblast proliferation in cardiac and pulmonary fibrosis [77, 78], and inhibition of ERK activity has been shown to attenuate lung injury and inflammation induced by bleomycin in a murine model [79]. Moreover, activation of ERK signaling is related to the presence of NOX and ROS [80]. NOX inhibitors have been shown to suppress the activation of ERK1/2 and EMT in human tubular epithelial cells, an effect that was mainly related to the reduction of ROS levels [81]. Activation of ERK signaling promotes the expression of CTGF, the proliferation of fibroblasts, and the deposition of ECM [82].

In addition to being associated with apoptosis, ROS are also involved in autophagy [83], an intracellular degradation pathway that plays a role in both normal physiological and pathological processes. In general, autophagy is a complex biological process that involves the initiation of the formation of phagophores and autophagosomes, the generation of lysosomes, autophagosome–lysosome fusion, and, finally, degradation. ROS exert dual effects in cells, as they are the basis of oxidative damage and are also present in normally functioning cells. A moderate increase in ROS levels can serve as a signal to induce autophagy, and there is evidence suggesting that if ROS production continues to increase, it may cause damage to the lysosomal membrane [84], which could affect autophagy. In recent years, studies have found that pulmonary fibrosis in lung tissue is accompanied by insufficient autophagy, which causes senescence and injury of AECs, facilitates EMT, and promotes differentiation of fibroblasts into myofibroblasts. Epithelial dysfunction and fibroblast proliferation are generally associated with impaired autophagy [85]. Therefore, the restoration of autophagy can inhibit fibroblast differentiation, reduce collagen deposition, and inhibit pulmonary fibrosis, and there is evidence to show that simvastatin reduces airway inflammation by upregulating autophagy in mouse models of asthma [86].

The expression of ROS is significantly upregulated in the lung tissues of patients with IPF, a change that may be related to external stimuli, pharmacological factors, and the continuous release of inflammatory cells. Increased apoptosis and inadequate autophagy have also been observed in the lung tissues of patients with IPF, and the changes are associated with the altered activity of ROS-mediated signaling pathways (see Figure 2). Thus, statins can interact with the ROS signaling pathways to exert antifibrotic effects.

### 2.4. Basic Science Studies Investigating the Effects of Statins on IPF

In 2004, Watts et al. found that simvastatin, which blocks Rho prenylation and its subsequent signaling, can significantly inhibit CTGF gene expression in normal human lung fibroblasts (IMR 90 cells) and IPF-derived lung fibroblasts (LL29, LL97a, and HIPF cells), modulate TGF-*β*/CTGF interactions, and specifically override the potent induction of CTGF by TGF-*β* [87]. Geranylgeranyl-pyrophosphate (GGPP) is an intermediate in the cholesterol synthesis pathway that can modify RhoA through a reaction catalyzed by isoprene transferase, a process known as Rho prenylation [88]. Statins can reduce GGPP synthesis by inhibiting the activity of HMG-CoA reductase, thereby reducing the membrane-bound fraction of RhoA in fibroblasts [89]. Rho protein and the actin cytoskeleton are considered the key determinants of TGF-*β*-induced CTGF expression, and loss of Rho protein can inhibit the expression of CTGF [90]. In summary, simvastatin inhibits the cholesterol synthesis pathway, a process that is associated with the inhibition of Rho prenylation and the blockade of the Rho signaling pathway, and inhibits the expression of CTGF genes and proteins in fibroblasts.

Ou et al. confirmed that simvastatin could reduce the number of neutrophils and lymphocytes, and inhibit the expression of TNF-*α* in the bronchoalveolar lavage fluid of mice, and it could also inhibit the expression of TGF-*β* and CTGF and reduce the accumulation of collagen in a murine model of bleomycin-induced pulmonary fibrosis [91]. The study also found a significant increase in the level of hydroxyproline in the lungs of mice treated with bleomycin and a significant decrease in the hydroxyproline levels in the lungs of patients treated with simvastatin. Moreover, the hydroxyproline concentration in the lungs of mice correlated with the dose of simvastatin administered. The antipulmonary fibrotic mechanism of simvastatin is also related to the inhibition of Smad2/3 phosphorylation and RhoA expression [91]. For example, Tulek et al. found that high doses of simvastatin (5 mg/kg) significantly inhibited the expression of IL-13 and TGF-*β* in the bronchoalveolar lavage fluid of rats. However, they found that simvastatin did not reduce the levels of hydroxyproline in the lungs of bleomycin-treated rats [92]. Yang et al. observed similar effects as those in a study conducted by Ou et al. in which simvastatin attenuated TGF-*β*1-induced EMT and inhibited Smad2/3 phosphorylation [93]. Zhu et al. found that atorvastatin was capable of inhibiting CTGF and ERK signaling, reducing the level of MDA and NO in the lung tissues, and inhibiting the expression of iNOS. They also found that atorvastatin could reduce the oxidative damage caused by bleomycin in the lung tissues of mice and attenuate the bleomycin-induced pulmonary fibrosis [94]. Hamblin et al. found that lovastatin inhibited the expression of macrophage inflammatory protein 1-*α* (MIP-1-*α*) and significantly reduced the number of fibrocytes and the degree of collagen deposition in the lung tissues of mice. They also found that compared with that of the placebo group, mice in the lovastatin group exhibited a 45% lower risk of death, which represented a significant survival advantage [95]. As discussed in the previous subsection describing the pathogenesis of IPF, the increased abundance of ROS resulting from an imbalance between redox reactions plays an important role in IPF. MDA is a marker of oxidative damage that is generated by ROS attacking lipid molecules in the body. Khodayar et al. found that the serum MDA and lung hydroxyproline levels were significantly increased in a model of paraquat-induced pulmonary fibrosis in rats, and the levels of both were significantly reduced by atorvastatin, alleviating pulmonary fibrosis [96]. ROS, TGF-*β*, and p38 MAPK interact with each other to jointly affect the degree of tissue fibrosis. In a study that investigated the effects of statins on acute hypoxia-induced fibroblast proliferation in the lungs and systemic arterial system and on p38 MAPK activity, Carlin et al. found that fluvastatin was effective in inhibiting both processes [97]. In another study, researchers found that simvastatin protected the endothelial barrier by inhibiting NOX activity and superoxide production [98]. El-Mohandes et al. found that amiodarone was capable of inducing the generation of degranulated mast cells and alveolar macrophages in alveolar sacs, and the administration of atorvastatin significantly reduced the number of mast cells and alveolar macrophages and inhibited pulmonary fibrosis in rats [99]. Mast cell granules contain histamine and TGF-*β*; following degranulation, the components can promote the proliferation of fibroblasts, and alveolar macrophages can also secrete TGF-*β*, thereby promoting the enhancement of collagen fiber synthesis and leading to the deposition of ECM [100]. In 2017, Lee et al. found that simvastatin was able to promote the antifibrotic properties associated with the early perfusion of apoptotic cells in the middle stage of bleomycin-induced pulmonary fibrosis in mice, and the combined action of simvastatin and the administration of apoptotic cells further enhanced the expression of PPAR-*γ* in alveolar macrophages and inhibited the pulmonary fibrotic response [101]. The beneficial effects of simvastatin on IPF are primarily achieved by enhancing the specific anti-EMT and antifibrotic properties of AECIIs and lung fibroblasts. YAP/TAZ is expressed in the nuclei of fibroblasts and mediates tissue fibrosis [102]. Studies have reported that the inhibition of YAP/TAZ inhibits fibroblast differentiation and reverses pulmonary fibrosis [103]. For example, Santos et al. found that simvastatin inhibits YAP activity through the mevalonate pathway, disrupts profibrotic fibroblast differentiation, and alleviates pulmonary fibrosis in mice [104]. The mevalonate pathway is responsible for the synthesis of isoprene compounds that are critical for cell growth, such as GGPP, which mediates Rho guanosine triphosphatases (GTPases) and, in turn, promotes YAP/TAZ activation [105]. Simvastatin can inhibit the activity of the rate-limiting enzyme HMG-CoA reductase in the mevalonate pathway, reducing the generation of GGPP and the activity of Rho GTPases, thereby affecting the activity of YAP/TAZ and causing YAP to become phosphorylated and degraded [46, 105].

In addition to these factors, researchers have found that there is a close relationship between cell senescence and IPF. Senescent cells can secrete a variety of cytokines, chemokines, growth factors, and MMPs, which constitute senescence-associated secretory phenotype (SASP) [106]. Minagawa et al. showed that TGF-*β* can induce senescence of the human bronchial epithelial cells, secrete excessive IL-1*β*, and promote the transformation of fibroblasts into myofibroblasts in the IPF lung samples [107]. Schafer et al. found that the senescent fibroblasts secreted a large amount of SASP, including TGF-*β*, interleukin-6 (IL-6), and MMP-12, which regulated pulmonary fibrosis, and deletion of senescent cells reduces pulmonary expression of these factors [108]. According to research, fibroblasts derived from lung biopsies of patients with IPF showed accelerated replicative cellular senescence [109]. Liu et al. found that simvastatin can significantly reduce the SASP of senescent human fibroblasts by inhibiting Rho prenylation and can also reduce the expression of IL-1*β*, IL-6, and TGF-*β* [110]. This indicates that simvastatin is an effective SASP inhibitor. Thus, it seems that the elimination of senescent cells and the blocking of SASP can provide a new therapeutic opportunity for this fatal disease.

Collectively, the basic science trials described above (and summarized in Table 1) have shown that statins can alleviate the inflammatory response, reduce lung tissue damage, inhibit the expression of cytokines through various mechanisms, suppress or block the signaling pathway that drives pulmonary fibrosis, reduce the proliferation of fibroblasts and the deposition of collagen in the lung, and, ultimately, inhibit the development of pulmonary fibrosis (see Figure 3).

### 2.5. Clinical Trials Investigating the Effects of Statins on IPF

The earliest clinical trial to investigate the association between IPF and the use of statins was published in 2004. A total of 477 participants diagnosed with IPF were included in the study, among whom 35 (7%) were treated with statins, 18 were with lovastatin, nine were treated with simvastatin, six with pravastatin, and two with fluvastatin; the remaining 442 (93%) participants were not treated with statins. The mean age of the patients in the statin group was 66.6 ± 8.7 years, whereas that in the nonstatin group was 70.9 ± 8.9 years. The study comprised 29 men (83%) in the statin group and 302 men (68%) in the nonstatin group. Nadrous et al. [111] retrospectively analyzed the data in 2004 and found that the median survival for both groups was 2.9 years, with or without statins. There was no significant difference in the median survival (hazard ratio (HR): 0.97 (95% confidence interval (CI): 0.62–1.52); *P* = 0.895) after adjusting for comorbidities due to the large variability in the baseline measurements between the two groups. The statistical results showed that the use of statins did not improve the median survival time of patients with IPF. Concurrently, researchers also found that the prevalence of coronary heart disease and the number of smokers were significantly higher in the statin group than in the control group, and the number of participants in the statin group was lower, which may explain the negative results of that study.

Despite the lack of effect, these findings did not discourage researchers from investigating whether statins are effective in the treatment of IPF. For example, in 2015, Vedel-Krogh et al. [112] retrospectively analyzed the clinical data of the entire Danish population diagnosed with interstitial pulmonary disease from 1995 to 2009. A total of 783 patients diagnosed with IPF were included in the study. The mean age at diagnosis of IPF was 73 years, with 261 patients in the statin group (33%) and 522 patients in the nonstatin group (67%). In terms of sex, 162 men (62%) were included in the statin group, and 324 men (62%) were included in the nonstatin group. The median survival times of the participants in the statin and nonstatin groups were 3.4 and 2.4 years, respectively. A significant difference in all-cause mortality was observed between the two groups (HR: 0.76 (95% CI: 0.62–0.93); *P* = 0.05), which suggested that the use of statins could prolong the median survival time of patients with IPF while also reducing the all-cause mortality.

However, the results of a prospective cohort study did not show reduced mortality in patients with IPF with the use of statins. A total of 462 patients (mean age: 76.5 ± 9.1 years) diagnosed with IPF and who had started long-term oxygen therapy were enrolled, including 312 men (68%) and 150 women (32%). There were 122 (26%) patients in the statin group and 340 (74%) in the nonstatin group. Ekstrom et al. [113] found no statistically significant difference in mortality between statin users and nonusers (HR: 1.13 (95% CI: 0.81–1.57)). This study included patients with severe IPF who received long-term oxygen therapy and who were older and had more comorbidities. In addition, approximately 329 (71%) of the patients died during the median observation period, making it somewhat difficult to interpret the study's findings.

In a post hoc analysis of statin treatment for IPF, 624 patients diagnosed with IPF were included, including 276 (44%) in the statin group and 348 (56%) in the nonstatin group. There were 465 men (75%) and 159 women (25%) in the study. The baseline characteristics were similar between the groups, except that the mean age was higher in the statin group than in the nonstatin group (68.2 ± 7.0 years vs. 66.3 ± 7.8 years, respectively), and the statin group had a higher risk of cardiovascular disease. Kreuter et al. [114] analyzed the effects of statins on disease progression, mortality (both IPF-related mortality and all-cause mortality), the distance traveled in the 6-minute walk test, lung function, and hospitalization rates in 2017. The results showed that there was no difference between the two groups in terms of disease progression (multivariate HR: 0.75 (95% CI: 0.52–1.07); *P* = 0.1135), all-cause mortality (multivariate HR: 0.54 (95% CI: 0.24–1.21); *P* = 0.1369) or absolute forced vital capacity (FVC) decrease ≥ 10% (multivariate HR: 0.71 (95% CI: 0.48–1.07); *P* = 0.1032). However, there were statistically significant differences between the group in terms of a decrease in the 6-minute walk distance of >50 m (multivariate HR: 0.69 (95% CI: 0.48–0.99); *P* = 0.0465), all-cause hospitalization (multivariate HR: 0.58 (95% CI: 0.35–0.94); *P* = 0.0289), respiratory-related hospitalization (multivariate HR: 0.44 (95% CI: 0.25–0.80); *P* = 0.0063), and IPF-related mortality (multivariate HR: 0.36 (95% CI: 0.14–0.95); *P* = 0.0393). The findings suggested that the use of statins could reduce the hospitalization rates, delay the decrease in the 6-minute walk distance, prolong the survival time, and improve the quality of life in patients with IPF.

Kreuter et al. [115] published another study on statin therapy for IPF in 2018. A total of 1,061 patients diagnosed with IPF within the previous 5 years were included in the study. There were 312 (29%) patients using statins at baseline (192 in the nintedanib group and 120 in the placebo group) and 749 (71%) patients who were not (446 in the nintedanib group and 303 in the placebo group). The mean ages of those in the statin and nonstatin groups were 68.6 ± 7.1 years and 66.0 ± 8.3 years, respectively. There were 249 men in the statin group (79.8%) and 592 men in the control group (79.0%). Except for the older age and higher risk of cardiovascular disease in the statin group, the clinical symptoms of the other subgroups were similar. A post hoc analysis of the data conducted by Kreuter et al. in 2018 found that the annual rate of FVC decline in lung function was lower at -187.4 mL/year in the placebo group that was receiving statins at baseline than the decline of -238.1 mL/year in the placebo group that was not receiving statins (difference: 50.8 mL/year (95% CI: -10.9–112.5); *P* = 0.1065), although the difference was not statistically significant. There was no statistically significant difference between the two groups in the decline in FVC% of ≥5% predicted or death (HR: 0.81 (95% CI: 0.62–1.06); *P* = 0.1235), decline in FVC% of ≥10% predicted or death (HR: 1.01 (95% CI: 0.72–1.41); *P* = 0.9700), time of the first acute exacerbation of IPF (HR: 0.76 (95% CI: 0.33–1.73); *P* = 0.5144), or the St. George's Respiratory Questionnaire (SGRQ) total score (difference: 1.22 (95% CI: -1.65–4.09); *P* = 0.4039). Studies have shown that statins do not improve IPF-related mortality or the first acute exacerbation, and although they may delay the decline in FVC, they cannot completely prevent the progressive decline of FVC. In 2018, Kreuter et al. also investigated whether using statins at baseline increased the antifibrotic effect of nintedanib; the results showed that compared with nintedanib alone, the use of nintedanib in combination with statins had no significant effects on FVC, SGRQ score, disease progression, or acute exacerbations in patients with IPF.

A recently published study included 323 patients diagnosed with IPF between January 2013 and December 2017, with an average age of 70.8 years at the time of IPF diagnosis. The study included 247 men (76.5%). In total, 171 patients (53%) were treated with statins (66 with atorvastatin, 52 with simvastatin, 36 with rosuvastatin, 16 with pravastatin, and one with fluvastatin) and 152 (47%) were not treated with statins during the study period. Lambert et al. [116] reported that the annual decrease in FVC was lower in the statin group than in the nonstatin group (-7.3% vs. -10.2%, respectively; 2.9% difference (95% CI: 1.6–4.4); *P* < 0.001), as was the decrease in annual diffusing capacity of the lungs for carbon monoxide (DLCO)(-4.2% vs. -5.5%, respectively; 1.3% difference (95% CI: 0.24–2.3), *P* = 0.013), but statins did not improve survival in patients with IPF (multivariate HR: 0.82 (95% CI: 0.50–1.35), *P* = 0.428). Lambert et al. also found that statins combined with nintedanib or pirfenidone did not improve lung function in patients with IPF compared with statins alone (FVC, *P* = 0.41 DLCO, *P* = 0.72).

The six clinical trials described above (and summarized in Table 2) were all published between 2004 and 2021. They included 3,730 participants in total, with more males than females, and 1,177 (32%) participants in the statin group. Among the six clinical trials, three were retrospective analyses, two were post hoc analyses, and one was a prospective cohort study. Three clinical trials examined the relationship between statin use and changes in FVC in patients with IPF. Kreuter et al. in 2018 and Lambert et al. in 2021 showed that statins could slow the decline of FVC in patients with IPF, and Lambert et al. also found that statins could delay the decline in lung function in terms of DLCO. However, in 2017, Kreuter et al. found that there was no correlation between the use of statins and FVC in patients with IPF. Studies by Vedel-Krogh et al. in 2015 and Kreuter et al. in 2017 showed that statins extended the median survival and reduced mortality in patients with IPF, whereas Nadrous et al. in 2004 and Ekstrom et al. in 2016 found that statins did not affect median survival in patients with IPF. In addition, in 2017, Kreuter et al. also found that statins significantly reduced IPF-related hospitalization and the decline in the 6-minute walk distance. In addition, Kreuter et al. in 2018 and Lambert et al. in 2021 found that statins combined with nintedanib or pirfenidone had little effect on lung function in patients with IPF, and that the combination did not enhance the antipulmonary fibrotic effects of the two drugs.

### 2.6. The Clinical Safety of Statins

Statins are commonly used to treat cardiovascular disease. Since receiving approval for marketing, this class of drugs has benefited countless patients with hyperlipidemia and coronary heart disease. In the existing clinical trials that have investigated the treatment of IPF with statins, there have been few reports on their side effects. Kreuter et al. [115] observed an incidence of diarrhea in 69.3% of patients receiving statins and 59.4% of patients not receiving statins taking nintedanib in 2018. However, approximately 62% and 60% of the subjects were treated with nintedanib in the statin and nonstatin groups, respectively, and the rate of serious adverse events was higher in the group that received nintedanib alone than that in the group that received combination therapy with nintedanib and statins. In a randomized, double-blind, phase III clinical trial investigating the efficacy and safety of nintedanib in the treatment of IPF, the researchers found that diarrhea was the main adverse effect; more specifically, in the Inpulsis-1 trial, 61.5% and 18.6% of patients in the nintedanib and placebo groups experienced diarrhea, respectively, whereas in the Inpulsis-2 trial, the incidence of diarrhea was 63.2% and 18.3% in the nintedanib and placebo groups, respectively [117]. Therefore, diarrhea can largely be attributed to the side effects of nintedanib, not of statins.

Thus, the benefits of statins outweigh the potential side effects, and the good clinical safety profile of this class of drugs makes them a potentially attractive option for the treatment of IPF.

## 3. Discussion

An increasing number of studies have shown that inflammation is the basis for the pathogenesis of IPF. In IPF, damage to lung tissue is mainly characterized by the infiltration of inflammatory cells, which can increase the expression of cytokines, activate NOX, promote the production of ROS, and mediate the mechanisms associated with injury, repair, and fibrosis. In the early stage of IPF, pulmonary vascular permeability increases, and the connections between the endothelial cells continue to open. This abnormal endothelial barrier function provides a bypass for macromolecule exchange and makes it possible for the inflammatory cells to enter the alveoli and interstitium during lung injury. IPF is a chronic progressive disease in which the normal physiological function of the alveolar tissue becomes impaired, affecting gas exchange and causing varying degrees of hypoxia. Patients eventually die due to respiratory failure; therefore, further studies on the pathogenesis and changes in related cytokines are crucial for the identification of novel therapeutic targets.

With the recent advances in metabolomics, researchers have observed changes in energy metabolism in patients with IPF. Understanding the effect of energy metabolism on the disease process will help deepen the understanding of the disease and possibly delay disease progression or even cure the disease by changing the energy metabolism pathway. Zhao et al. reported downregulation of the sphingolipid metabolism and upregulation of arginine metabolism, as well as changes in the metabolism of energy substances such as glucose and fatty acids in patients with IPF [118]. Sphingolipids and their metabolites sphingosine-1-phosphate (S1P) play key roles in inflammation, angiogenesis, endothelial barrier integrity, cell proliferation, differentiation, and migration and are regulators of cancer, fibrosis, and other diseases [119]. Studies have shown that S1P can enhance the endothelial barrier function and play a protective role in various acute lung injury models due to its ability to limit vascular leakage in the early stage of lung injury [120]. In the murine radiation-induced lung injury model, simvastatin reduced the infiltration of inflammatory cells and lung vascular leak, which was associated with changes in the sphingolipid metabolism [120]. Simvastatin can enhance the expression of barrier-promoting S1P receptor 1 (S1PR1) and enhance the endothelial barrier function, thus playing a protective role in the initial stage of inflammation [121]. In serum metabolic profiling, researchers found that the lysophosphatidylcholine (LysoPC) levels were two times more abundant in the serum of IPF patients compared to that of healthy participants [122]. It has been found that lysophosphatidic acid (LPA) levels increase in bronchoalveolar lavage fluid in a mouse model of bleomycin-induced pulmonary fibrosis [123]. The activation of LPA receptor LPA1 is associated with vascular leakage and increased fibroblast aggregation [123].

Studies have found that patients with IPF often experience different comorbidities. In a retrospective analysis of 272 patients diagnosed with IPF, researchers found that approximately 58% had one to three comorbidities, 30% had four to seven comorbidities, and only 12% had none; among these, cardiovascular comorbidities had the greatest impact on the mortality of patients with IPF [124]. Other studies have found that IPF is often complicated by pulmonary arterial hypertension, the incidence of which is as high as 86%. The discovery and treatment of these complications could help improve the quality of life and extend the survival of patients with IPF [125]. One study found that statins protected against pulmonary hypertension by reducing the severity of certain measures and slowing the progression of the disease, with pravastatin exerting the most significant effects [126]. Patients with IPF often experience complications due to cardiovascular diseases and pulmonary hypertension, which makes the use statins possible in patients with IPF.

Currently, statins are classified into two categories, natural compounds (simvastatin, lovastatin, and pravastatin) and synthetic compounds (atorvastatin, rosuvastatin, and fluvastatin) [127] (see Figure 4). The mechanism of action of statins is roughly the same, but the physicochemical properties and pharmacokinetics of statins are different. Simvastatin, lovastatin, and pravastatin are inhibitors of HMG-CoA reductase derived from fungal metabolites and have elimination half-lives of 1–3 hours [128]. Atorvastatin, rosuvastatin, and fluvastatin are synthetic compounds with elimination half-lives ranging from 1 to 19 hours [128]. Atorvastatin, simvastatin, lovastatin, and lovastatin are lipophilic compounds. Pravastatin and rosuvastatin are hydrophilic compounds [129]. Statins provide beneficial regulation of low-density lipoprotein cholesterol (LDL-C), high-density lipoprotein cholesterol (HDL-C), and triglycerides [129]. Simvastatin is a prodrug that is rapidly hydrolyzed into active metabolites, mainly *β*-hydroxyacid-simvastatin, which has a strong inhibitory effect on HMG-CoA reductase [130]. The study found that patients with hypercholesterolemia who received orally simvastatin 10 to 40 mg/day reduced plasma total cholesterol and LDL-C concentrations by 30 to 45% [130] and increased HDL-C concentrations by 5 to 15% [131]. Lovastatin is the first competitive inhibitor of HMG-CoA reductase, which inhibits cholesterol synthesis, decreases apolipoprotein B concentration, and increases LDL receptor activity [132]. Lovastatin is converted to a variety of active metabolites, primarily *β*-hydroxyacid-lovastatin [132]. The study found that the concentration of serum total cholesterol and LDL-C in patients with hyperlipidemia could be reduced by 25-40% after taking lovastatin 20 to 40 mg twice daily [132]. Pravastatin inhibits hepatic cholesterol synthesis and stimulates LDL receptor synthesis and activity, thereby reducing LDL-C levels [133]. The study found that patients with hypercholesterolemia who received pravastatin 5 to 20 mg twice daily reduced LDL-C concentrations by 18 to 31% [133]. Atorvastatin can inhibit HMG-CoA reductase and the formation of mevalonic acid, thereby reducing serum cholesterol and LDL-C levels [134]. Patients with hypercholesterolemia who received atorvastatin 10 to 80 mg/day reduced LDL-C concentrations by 35 to 60% [134]. Rosuvastatin has a high affinity for the active site of HMG-CoA reductase activity and strong inhibition of HMG-CoA reductase and cholesterol synthesis, making it the most effective at lowering LDL-C [135]. Patients with hypercholesterolemia who received fluvastatin 20 or 40 mg/day reduced LDL-C concentrations (19 to 31%), total cholesterol levels (15 to 21%), triglyceride levels (1 to 12%), and increased HDL-C concentrations (2-10%) [136]. Different statins can be used to reduce cholesterol synthesis in the liver; however, the specific effects of various types of statins in IPF remain unclear.

On reviewing the literature, we noted that Xu et al. reported that statins can aggravate pulmonary fibrosis. In their regression analysis, researchers found that statin use was associated with interstitial lung abnormalities among smokers and that statins enhance bleomycin-induced lung inflammation and fibrosis in mice through a mechanism involving enhanced NOD-, LRR-, and pyrin domain-containing protein 3 (NLRP3) inflammasome activation, which appears to be related to the increase in mitochondrial ROS associated with the administration of statins [137]. Similarly, Larson-Casey et al. reported that simvastatin promoted pulmonary fibrosis by increasing the RAS-related C3 botulinum substrate 1 (Rac1) activity in macrophages, which was associated with the Akt1 signaling pathway [138]. These results appear to contradict the findings raised in our previous discussion of the antifibrotic properties of statins, the exact mechanism of which remains unclear.

It has been demonstrated that statins can inhibit the inflammatory response after lung tissue injury, reduce the number of inflammatory cells, decrease the expression of TGF-*β*/CTGF, inhibit the Rho signaling pathway and the phosphorylation of Smad2/3, suppress the activity of YAP/TAZ, and attenuate pulmonary fibrosis in basic science studies, including *in vitro* assays or animal models. In clinical trials in humans, Kreuter et al. in 2018 and Lambert et al. in 2021 showed that statins could slow the decline in FVC in patients with IPF, and Lambert et al. also found that statins could delay the decline of lung diffusion capacity. Vedel-Krogh et al. in 2015 and Kreuter et al. in 2017 showed that statins extended the median survival time and reduced mortality in patients with IPF, with the study by Kreuter et al. also showing that statins significantly reduced IPF-related hospitalizations and delayed the decrease in the 6-minute walk distance. Collectively, these clinical trials demonstrated the possibility that statins could be efficacious in the treatment of IPF. However, some findings have been negative or contradictory; for example, Kreuter et al. in 2017 showed that statins did not delay the decline in FVC in patients with IPF, and Nadrous et al. and Ekstrom et al. found that statins did not prolong the median survival time of patients with IPF. Lung function is closely related to age and individual baseline conditions, such as cardiovascular diseases and hyperlipidemia, which may lead to impaired lung function [139]. The negative results of those clinical trials may have been due to the patients in the statin group being older, on average, and having more complicated cardiovascular diseases at baseline, which would have affected the pulmonary function and survival rate of patients with IPF. It is also possible that the results were biased due to the small number of participants in the statin group.

To date, only two drugs have been approved for the treatment of IPF, including nintedanib and pirfenidone. Nintedanib (formerly known as BIBF1120) is a potent intracellular inhibitor of tyrosine kinases that competitively binds to the kinase domains of vascular endothelial growth factor (VEGF), platelet-derived growth factor (PDGF), and fibroblast growth factor (FGF) [140]. In a randomized, double-blind phase III clinical trial conducted over a period of 52 weeks, nintedanib significantly delayed the decline in lung function [117]. Pirfenidone is a synthetic molecule with high bioavailability that regulates the activation of TGF-*β* and inhibits the proliferation of fibroblasts [141]. In a clinical study that investigated the efficacy of pirfenidone in the treatment of IPF, pirfenidone reduced the decline in FVC (*P* = 0.001) and was more effective at 24 weeks compared with the placebo group, but there was no difference in the percentage of predicted DLCO or dyspnea [142]. In another clinical study, pirfenidone reduced the decrease in the 6-minute walk distance compared with that in the control group, and, most importantly, it reduced mortality in those with IPF. Common adverse drug reactions included gastrointestinal symptoms, and 14.4% of patients discontinued the medication due to adverse drug reactions, while three patients gradually deteriorated [143]. According to the results, nintedanib and pirfenidone were capable of delaying the decline in FVC, and the pirfenidone also reduced mortality in patients with IPF. In 2018, Kreuter et al. investigated whether the use of statins at baseline increased the efficacy of nintedanib and found no improvement in lung function in terms of FVC, SGRQ score, disease progression, or acute exacerbation compared with nintedanib. Lambert et al. found that statins combined with nintedanib and pirfenidone had little effect on lung function in patients with IPF and did not enhance the antifibrotic effect of the two drugs. Given the differences in the baseline characteristics of the populations included in the clinical trials, the relative safety and low cost of statins, and the previous basic science and clinical studies that have demonstrated the efficacy of statins as a potential treatment for IPF, the efficacy of statins in the treatment of IPF should be reassessed.

## 4. Conclusion

To date, basic science and clinical trials that have assessed the treatment of IPF with statins have predominantly focused on simvastatin and atorvastatin. The effects of various other types of statins on the treatment of IPF are unknown, and it is unclear whether different types of statins or those with a particular structure could have different benefits in patients with IPF. To date, no prospective, randomized, controlled, double-blind trials have been conducted to evaluate the efficacy of statins in the treatment of IPF. More clinical studies are required to determine the efficacy of statins alone in the treatment of IPF and its related comorbidities; in addition, we hope to determine whether combination treatments with statins and the currently available antipulmonary fibrosis drugs such as nintedanib and pirfenidone would benefit patients with IPF compared with the administration of statins alone. We hope to focus on the research and development of molecular targeted therapies to delay the progression of the disease and improve the survival rate and quality of life in patients with IPF.

## Figures and Tables

**Figure 1:** TGF-*β* is a multifunctional cytokine that regulates cell growth and differentiation. TGF-*β* binds to receptors (including T*β*R-I and T*β*R-II) at the cell membrane and promotes fibrosis through the activation of Smad and Smad-independent signaling pathways. The cell signaling pathways involved in pulmonary fibrosis mainly include TGF-*β*/Smad, TGF-*β*-Ras-Raf-MEK-ERK1/2, TGF-*β*-TAK1/TAB1-MKK3-p38, and TGF-*β*-TAK1/TAB1-MKK4-JNK. Abbreviations: ERK: extracellular signal-regulated kinase; Grb2: growth factor receptor-bound protein 2; JNK: c-Jun N-terminal kinase; MEK: mitogen-activated protein kinase kinase; MKK3: mitogen-activated protein kinase kinase 3; MKK4: mitogen-activated protein kinase kinase 4; p38: p38 mitogen-activated protein kinase; Sos: Son of Sevenless; TAB1: TAK1 binding protein 1; TAK1: TGF-*β*-activated kinase 1; TGF-*β*: tumor growth factor beta; T*β*R-I: TGF-*β* receptor type I; T*β*R-II: TGF-*β* receptor type II.

**Figure 2:** A schematic showing some mechanisms through which ROS may disrupt processes related to autophagy and apoptosis. External stimuli, pharmacological factors, and inflammatory cells can lead to upregulated levels of ROS, resulting in autophagy and apoptotic dysfunction of cells in lung tissues. ROS can mediate increased apoptosis of the lung epithelial cells through endoplasmic reticulum stress, changes in mitochondrial and p38/JNK/ERK signaling, and insufficient fibroblast autophagy resulting from lysosomal membrane injury. Collectively, these factors contribute to pulmonary fibrosis. Abbreviations: Bcl-2: B-cell lymphoma 2; Bax: B-cell lymphoma 2-associated X protein; ER: endoplasmic reticulum; ERK: extracellular signal-regulated kinase; JNK: c-Jun N-terminal kinase; NADPH: nicotinamide adenine dinucleotide phosphate; p38: p38 mitogen-activated protein kinase; ROS: reactive oxygen species.

**Figure 3:** A summary of the mechanisms through which statins attenuate pulmonary fibrosis. Inflammatory cells release inflammatory factors and the profibrotic factor TGF-*β*, which promote ROS release and activate ROS-related signaling pathways. Statins inhibit inflammation and act on ROS-related signaling pathways. In addition, statins upregulate PPAR-*γ* expression, which inhibits the activity of TGF-*β*, as well as YAP activity through the mevalonate pathway. Statins inhibit TGF-*β* and CTGF expression in fibroblasts by inhibiting the cholesterol synthesis pathway, which is associated with the inhibition of Rho prenylation. Abbreviations: CGTF: connective tissue growth factor; ECM: extracellular matrix; ERK: extracellular signal-regulated kinase; GGPP: geranylgeranyl-pyrophosphate; HMG-CoA: 3-hydroxy-3-methylglutaryl-coenzyme A; IL-13: interleukin 13; NOX: nicotinamide adenine dinucleotide phosphate oxidase; p38: p38 mitogen-activated protein kinase; PPAR-*γ*: peroxisome proliferator-activated receptor gamma; Rho: Rho guanosine triphosphate-activating protein (GTPase); RhoA: transforming protein RhoA (Ras homolog family member A); ROS: reactive oxygen species; TGF-*β*: tumor growth factor beta; YAP: Yes-associated protein.

**Figure 4:** Examples of the chemical structures of various statins, including natural compounds (simvastatin, lovastatin, and pravastatin) and synthetic compounds (atorvastatin, rosuvastatin, and fluvastatin).

**Table 1:** Basic science trials investigating the effects of statins on IPF.

	Year	Model	Statin/Route of administration	Duration	Outcomes	Ref.
Watts et al.	2004	Normal human lung fibroblasts (IMR 90 cells) and IPF-derived lung fibroblasts (LL29, LL97a, and HIPF cells)	Simvastatin/-	-	Inhibited expression of TGF-*β* and CTGF Blocked Rho prenylation and Rho signaling pathways	[87]
Carlin et al.	2007	Fibroblasts from adult male Sprague Dawley rats	Fluvastatin/-	-	Inhibited the proliferation of fibroblasts Inhibited p38 MAPK activity	[97]
Chen et al.	2008	Human pulmonary artery endothelial cells	Simvastatin/-	-	Inhibited NOX activity and superoxide production	[98]
Ou et al.	2008	C57BL/6 mice (bleomycin-induced pulmonary fibrosis)	Simvastatin/ intratracheal injection	7 or 28 days	Reduced the number of neutrophils and lymphocytes Inhibited the expression of TNF-*α* Decreased the expression of TGF-*β* and CTGF Decreased lung collagen accumulation Inhibited Smad2/3 phosphorylation Inhibited expression of RhoA	[91]
Tulek et al.	2012	Female Sprague Dawley rats (bleomycin-induced pulmonary fibrosis)	Simvastatin/-	14 days	Decreased the expression levels of IL-13 and TGF-*β*	[92]
Yang et al.	2013	A549 cell line	Simvastatin/-	-	Suppressed Smad2/3 phosphorylation Decreased TGF-*β*1-induced EMT	[93]
Zhu et al.	2013	Male Sprague Dawley rats (bleomycin-induced pulmonary fibrosis)	Atorvastatin/ intragastric administration	28 days	Inhibited CTGF and ERK signaling pathways Reduced the levels of MDA and NO expression Suppressed the expression of iNOS	[94]
Hamblin et al.	2014	C57BL/6 mice (bleomycin-induced pulmonary fibrosis)	Lovastatin/ oral administration	8 or 14 days	Inhibited the expression of MIP-1-*α* Reduced the number of fibrocytes Decreased lung collagen accumulation Reduced the risk of death in mice	[95]
Khodayar et al.	2014	Female Sprague Dawley rats	Atorvastatin/ oral administration	21 days	Reduced hydroxyproline content Reduced serum MDA level	[96]
Liu et al.	2015	Normal human fibroblasts HCA2	Simvastatin/-	-	Reduced the SASP of senescent human fibroblasts Reduced the expression of IL-1*β*, IL-6, and TGF-*β* Blocked Rho prenylation	[110]
El-Mohande et al.	2017	Male albino rats (amiodarone)	Atorvastatin/ oral administration	3 months	Decreased the number of mast cells and alveolar macrophages	[99]
Lee et al.	2017	Mice (bleomycin-induced pulmonary fibrosis)	Simvastatin/-	-	Increased the expression of PPAR-*γ*	[101]
Santos et al.	2020	Mice (bleomycin-induced pulmonary fibrosis)	Simvastatin /-	-	Suppressed activation of YAP	[104]

Abbreviations: CTGF: connective tissue growth factor; EMT: epithelial-mesenchymal transformation; ERK: extracellular signal-regulated kinase; IL-1*β*: interleukin 1*β*; IL-6: interleukin 6; IL-13: interleukin 13; iNOS: inducible nitric oxide synthase; MDA: malondialdehyde; MIP-1-*α*: macrophage inflammatory protein 1-*α*; NO: nitric oxide; NOX: nicotinamide adenine dinucleotide phosphate oxidase; p38 MAPK: p38 mitogen-activated protein kinase; PPAR-*γ*: peroxisome proliferator-activated receptor gamma; RhoA: transforming protein RhoA (Ras homolog family member A);SASP: senescence-associated secretory phenotype; TGF-*β*: tumor growth factor beta; TNF-*α*: tumor necrosis factor alpha; YAP: Yes-associated protein.

**Table 2:** The clinical trials that have investigated the effects of statins on IPF.

	Year	Differential intervention in study groups	Sex ratio (male/female)	Age (years)	Sample size (N)	Number of statin users	Outcomes	Ref.
Nadrous et al.	2004	Statin vs. Never user	S: 29/6 C: 302/140	S: 66.6±8.7 C: 70.9±8.9	477	35	Median survival time	[111]
Vedel-Krogh et al.	2015	Statin vs. Never user	S: 162/99 C: 324/198	-	783	261	Median survival time All-cause mortality	[112]
Ekstrom et al.	2016	Statin vs. Antacid/*β*-blocker/diuretic	312/150	76.5±9.1	462	122	Mortality rate	[113]
Kreuter et al.	2017	Statin+ Placebo vs. Placebo	S: 225/51 C: 240/108	S: 68.2±7 C: 66.3±7.8	624	276	Disease progression Mortality (all-cause/IPF-related) Decrease in the 6MWD > 50 m Hospitalization (all-cause/respiratory-related)	[114]
Kreuter et al.	2018	Statin (nintedanib+ placebo) vs. Never user (nintedanib+ placebo)	S: 249/63 C: 592/157	S: 68.6±7.1 C: 66.0±8.3	1061	312	Annual rate of decline in FVC Decline in FVC% ≥ 5%/10% predicted or death Time of the first acute exacerbation of IPF SGRQ total score	[115]
Lambert et al.	2021	Statin vs. Never user	247/76	-	323	171	Annual FVC decline Annual DLCO decline	[116]

Abbreviations: 6MWD: 6-minute walk distance; C: control group; DLCO: diffusing capacity of the lungs for carbon monoxide; FVC: forced vital capacity; IPF: idiopathic pulmonary fibrosis; SQRQ: St. George's Respiratory Questionnaire; S: statin group.

## Data Availability

Not applicable.
